The article "A BP Neural Network Algorithm for Multimedia Data Monitoring of Air Particulate Matter" was published in 2022. Journal: Comput Intell Neurosci.

# A BP Neural Network Algorithm for Multimedia Data Monitoring of Air Particulate Matter

**DOI:** 10.1155/2022/6393877

**Published:** 2022-05-31

**Authors:** Chunyi Zhang

**Affiliations:** ^1^School of Environmental Science & Engineering, Tianjin University, Tianjin 300072, China; ^2^Tianjin Research Institute for Water Transport Engineering, M.O.T., Tianjin 300456, China

## Abstract

In order to study a BP neural network algorithm for air particulate matter data monitoring, firstly, the monitoring data collected by particle sensor using the light scattering method are proposed. Then, based on the improved BP neural network method, the mapping relationship between the actual measured value of the sensor, weather and other influencing factors, and the standard value of the monitoring station is established, and the calibration model of air particulate matter is realized. Finally, through theoretical analysis and experimental comparison, the results show that the model based on BP neural network algorithm has good accuracy and generalization ability in the evaluation of air particulate index, which makes it possible to scientifically and accurately refine the evaluation and management of urban air particulate index. The experimental results show that the air particle calibration model based on the light scattering method and improved BP neural network algorithm is practical and effective.

## 1. Introduction

Air is the “life gas” that human beings breathe every day and a necessary condition for our survival on the Earth. Therefore, the quality of air will directly affect our quality of life. With the continuous progress and development of human society, the rapid increase of urban population, and the sharp increase of the number of motor vehicles in China, the environmental pollution of our life is becoming more and more serious. The main source of PM_2.5_ is the residues discharged from combustion in the process of daily power generation, industrial production, and vehicle exhaust emissions, most of which contain toxic substances such as heavy metals. Generally speaking, coarse particles with a particle size of 2.5 microns to 10 microns Mainly from road dust, etc., fine particulate matter (PM_2.5_) below 2.5 microns mainly comes from the combustion of fossil fuels (such as motor vehicle exhaust and coal burning), volatile organic compounds, etc. (Figure 1), soil pollution, and other pollution; air pollution has become more and more serious. With the deterioration of air quality, the phenomenon of cloudy weather is increasing and the harm is aggravating [1]. In many parts of China, Yin Ting weather phenomenon is incorporated into fog as a disastrous weather early warning forecast, which is collectively referred to as “fog Ting weather.” Smog is a state of air pollution. Smog is a general expression of the excessive content of various suspended particles in the atmosphere, in which PM_2.5_ is considered to be the “culprit” of smog. At the beginning of 2013, fog and thunder swept the whole Middle East of China, among which Beijing Tianjin Hebei region was the most polluted, and the daily average fine particle PM_2.5_ concentration was as high as 500 *μ*g/m^3^. Since then, the pollution of PM_2.5_ has been widely concerned by the society. In recent years, PM_2.5_ has gradually become the primary pollutant of air pollution and an important standard for people to evaluate air quality. There are many kinds of antifog masks, air purifiers, and other products on the market.

The article "A BP Neural Network Algorithm for Multimedia Data Monitoring of Air Particulate Matter" was published in 2022. Journal: Comput Intell Neurosci.

The impact of PM_2.5_ on people's life is obvious to all, so the concentration of particulate matter in the air has become an indispensable air quality index in human daily life. It is urgent to monitor the concentration of particulate matter in the air and further use the monitored historical data to predict the concentration of particulate matter in a certain period of time in the future. However, the prediction of PM_2.5_ concentration is not easy. Compared with the conventional weather forecast, the weather condition forecast of air pollution not only needs the weather element data but also the air composition data is very important. However, the collection and acquisition of pollution source data are not easy. Many pollution sources change constantly in the process of pollution, and the data are always in the process of updating. At the same time, the prediction of PM_2.5_ concentration requires high accuracy of near stratum meteorological data, and the near stratum is affected by factors such as ground roughness, vegetation, and urban heat island effect, and the numerical deviation is large. In addition, in order to accurately predict the concentration of PM_2.5_, it is necessary not only to have an accurate understanding of the physical and chemical mechanism of PM_2.5_ but also to obtain the basic data of ground pollution sources, that is, the pollutant emission list, to do the application research of numerical prediction. When forecasting, we should be able to understand the interaction and law of the two processes, coupled with experience, in order to make an accurate forecast, which is a very difficult work.

In a word, each urban environment is a complex large-scale system with the characteristics of high dimension, multivariable, complex relationship between influencing factors, and poor information integrity. It will take a long time to make the forecast directly. However, for such complex data processing, using artificial neural network to predict is a good choice. Artificial neural network is a model of human brain neural network. Its biggest feature is that it has strong nonlinear computing ability. Artificial neural network can build a model through the characteristics of input and output data [2]. In practical modeling, artificial neural network has good expansibility. We can optimize the network through various methods to improve the prediction accuracy of neural network. Artificial neural network is not single. We can flexibly build a specific network according to the specific situation of the city. Because of these characteristics of artificial network, artificial neural network has also been widely used in the prediction of air pollutants. Compared with traditional physical prediction methods, artificial neural network can predict the concentration of air particulate matter more quickly, conveniently, and accurately.

The article "A BP Neural Network Algorithm for Multimedia Data Monitoring of Air Particulate Matter" was published in 2022. Journal: Comput Intell Neurosci.

In this study, based on BP neural network algorithm, the air particulate matter values and other atmospheric-related eigenvalues collected by low-cost light scattering sensor are trained and learned, so as to establish the model mapping between eigenvalues and air particulate matter index at national control points, and then, use this model to convert eigenvalues into standard air particulate matter index. It provides an idea for realizing the high-density grid deployment of air monitoring equipment.

## 2. Literature Review

Wang et al. used the principal component analysis method to reduce the dimension of the original data and generated a new set of linear combinations using the original data as the input parameters of the neural network. The results show that the data obtained after the principal component analysis are more conducive to the learning of the neural network and improve the prediction accuracy of the neural network [3]. Guo et al. used the sensitivity algorithm to calculate the sensitivity between each parameter and PM_2.5_ and selected the parameters with high sensitivity as the input parameters of the whole neural network. The idea of this method is similar to that of principal component analysis, which can reduce the redundant input parameters, so as to reduce the training difficulty of neural network. It also helps the neural network to learn the functional relationship between the input parameters more easily and finally achieve the purpose of improving the prediction accuracy of the neural network [4]. Wen et al. did not use genetic algorithm to optimize the initial value of neural network weight, but used genetic algorithm to screen the input parameters of neural network. The parameters selected by researchers can be better learned by neural network, so the effect of neural network training is better, and the final prediction result is more accurate. The above is the optimization research on the input parameters of neural network [5]. Chen et al. combined K-means clustering algorithm with neural network to establish a new neural network model, which improved the prediction accuracy of neural network for PM_2.5_ and PM_10_ concentration values [6]. Liu et al. proposed a hybrid model combining artificial neural network and chaotic particle swarm optimization algorithm to improve the prediction accuracy. Chaotic particle swarm optimization algorithm is a search algorithm based on chaos, which can well identify nonlinear patterns [7]. Li et al. divided a variety of prediction factors into many individual prediction results through wavelet transformation algorithm and then synthesized these result sets into the final prediction results through neural network. The research results show good overall prediction accuracy. These algorithms can make up for some defects of neural network in the calculation process. Compared with the original neural network, the optimized neural network can predict the air quality more accurately. In terms of model combination, researchers skillfully combined the neural network model with other models to establish a new neural network model. The new neural network model can effectively improve the prediction accuracy of neural network [8]. Mahajan et al. combined the nearest neighbor model with the artificial neural network model. The input of the model is the concentration measured in several monitoring stations distributed in the whole city and the meteorological information in the area. At the same monitoring station, the expected maximum concentration is used as the output of the next day. The results show that the model may be considered as an important tool for air pollution control [9]. Blagojevi et al. combined the nearest neighbor model with the artificial neural network model. The input of the model is the concentration measured in several monitoring stations distributed in the whole city and the meteorological information in the area. At the same monitoring station, the expected maximum concentration is used as the output of the next day. The results show that the model may be considered as an important tool for air pollution control [10].

The article "A BP Neural Network Algorithm for Multimedia Data Monitoring of Air Particulate Matter" was published in 2022. Journal: Comput Intell Neurosci.

## 3. Monitoring Method Based on the Light Scattering Method and Improved BP Neural Network Algorithm

Taking advantage of the advantages of the light scattering method in the monitoring of airborne suspended particles and combining with BP neural network algorithm to make up for the shortcomings of the light scattering method, a compact microambient air monitoring system with low cost and multiparameter integration with high-density grid layout can be realized. The grid monitoring system can fully cover the area and realize air pollution monitoring with high temporal and spatial resolution. Combined with the application of information-based big data, realize the functions of pollution source tracking, early warning, and prediction and provide more timely and effective decision support for environmental pollution prevention and control [11].

### 3.1. Light Scattering Method

The principle of measuring mass concentration by the light scattering method is based on the scattering theory of particles. When light shines on particles suspended in the air, scattered light is generated [12]. Under the condition of certain properties of particles, the scattered light intensity of particles is directly proportional to the particle size. By measuring the intensity of scattered light, the particles with different particle sizes can be counted, and then, the mass concentration of particles can be obtained by using the conversion coefficient. The light scattering method is widely used in real-time monitoring because of its fast speed, good stability, and small volume. The light scattering method is related to the refractive index of particles, the morphology of particles, and their components. The humidity in the atmosphere may be the main factor affecting these aspects. If the mass concentration of particulate matter in the atmosphere is measured in a certain humidity environment, the measurement results should not be ideal and will produce a certain degree of error. If we want to get ideal measurement results, we need to eliminate the influence of humidity on mass concentration [13].

### 3.2. BP Neural Network Algorithm

BP neural network is an artificial neural network realized by BP algorithm. Artificial neural network is an operation model inspired by the mechanism of resting and action potential of natural neurons. Neurons receive signals through synapses located on cell membranes or dendrites. When the received signal is large enough (exceeding a certain threshold), the neuron is activated and then transmits a signal through the axon. The transmitted signal may be accepted by another synapse and may activate other neurons [14–17]. The physiological structure of the neuron is shown in Figure 2.

The artificial neuron model has made a highly abstract symbolic generalization of the complexity of natural neurons. The neuron model basically includes multiple inputs (similar to synapses). These inputs are multiplied by different weights (the received signal strength is different) [18] and then used by a mathematical function to calculate and decide whether to activate the neuron. This function is called the activation function, as shown in Figure 3. Artificial neural network combines these artificial neurons to process information. The greater the weight, the greater the influence of the input signal on neurons. The weight can be negative, which means that the input signal is suppressed. If the weights are different, the calculation of neurons is also different. By adjusting the weight, the required output value under fixed input can be obtained. The process of adjusting weights is called “learning” or “training” [19].

The article "A BP Neural Network Algorithm for Multimedia Data Monitoring of Air Particulate Matter" was published in 2022. Journal: Comput Intell Neurosci.

Based on the theoretical basis that the neural network algorithm can construct any complex function, we can establish a specific neural network model and use the sensor data collected by the light scattering method as the eigenvalue, and the data of the corresponding national control point or provincial control point as the feature label for training constantly adjust the weight of the network model and fit a corresponding function. Then, use this function for calibration. At the same time, considering the influence of environmental humidity on the light scattering method, the two eigenvalues of temperature and humidity need to be added to the training data so that the trained model will be more accurate. BP algorithm is the most commonly used and effective algorithm for training artificial neural network [20]. The neural network based on BP algorithm can learn and store a large number of input-output mode mapping relationships without revealing the mathematical equations describing this mapping relationship in advance. Its learning rule is to use the steepest descent method and continuously adjust the weight and threshold of the network through backpropagation. Its essence is to solve the minimum value problem of the error function. The specific process is as follows: randomly initialize the network weight and the threshold of neurons. Forward propagation: input the training set data into the input layer, pass through the hidden layer, finally reach the output layer and output the results, and calculate the input and output of hidden layer neurons and output layer neurons layer by layer according to the formula. Suppose the number of nodes in the input layer is *n*, the number of nodes in the hidden layer is *l*, and the number of nodes in the output layer is *m*. Suppose the number of nodes in the input layer is *n*, the number of nodes in the hidden layer is *l*, and the number of nodes in the output layer is *m* [21]. Input layer to hidden layer weight is *ω*_*i*_*j*__, hidden layer to output layer weight is *ω*_*jk*_, input layer to hidden layer offset is *a*_*j*_, hidden layer to output layer offset is *b*_*k*_, the learning rate is *η*, and the excitation function is *g*(*x*). The excitation function is Sig − moid function. The form is

(1) $$\begin{array}{c} g\left(x\right)=\frac{1}{1+e^{-x}}. \end{array}$$

The output of hidden layer *H*_*j*_ is

(2) $$\begin{array}{c} H_{j}=g\left(\sum_{i=1}^{n}\omega_{ij}x_{i}+a_{j}\right). \end{array}$$

Output of the output layer is

(3) $$\begin{array}{c} O_{k}=\sum_{j=1}^{l}H_{j}\omega_{jk}+b_{k}. \end{array}$$

Calculation formula of error is

(4) $$\begin{array}{c} E=\frac{1}{2}\sum_{k=1}^{m}{\left(Y_{k}-O_{k}\right)}^{2}, \end{array}$$

where *Y*_*k*_ is the desired output. If *Y*_*k*_ − *O*_*k*_=*e*_*k*_, it can be expressed as

(5) $$\begin{array}{c} E-\frac{1}{2}\sum_{k=1}^{m}c_{k}^{2}, \end{array}$$

where *i*=1 … *n*, *j*=1 … 1,  and *k*=1 … *m*.

The article "A BP Neural Network Algorithm for Multimedia Data Monitoring of Air Particulate Matter" was published in 2022. Journal: Comput Intell Neurosci.

Backward propagation: due to the error between the output result and the actual result, the error between the estimated value and the actual value is calculated, and the error is backpropagated from the output layer to the hidden layer until it is propagated to the input layer. The weight and threshold are modified according to the formula, and the above process is iterated continuously until the cumulative error of the training set meets the termination condition [12].

### 3.3. Improvement of BP Neural Network Algorithm

Before training data, we need to standardize the data and then use the standardized data for training. Different eigenvalue dimensions and dimensional units are also different, which will affect the training process and even the results. The standardized processing of data can eliminate the dimensional influence between indicators, so as to solve the comparability of eigenvalues. The BP neural network training data used in this study include four dimensions: PM_2.5_, PM_10_, humidity, and temperature. There is a large order of magnitude difference between each dimension. Direct training will lead to different gradient decline in each dimension. It is difficult to iterate to the lowest point of the cost function with the same learning rate. After normalization, the cost function becomes “rounder,” which makes it easy to reduce the gradient and improve the training speed. Common normalization methods include maximum minimum standardization, *Z* − Score standardization, and function transformation. Here, the maximum minimum standardization is used to linearly transform the original data. Let min*A* and max*A* be the minimum and maximum values of *A*, respectively, and map an original value *x* of *A* to the value *x*′ of interval [0,1] through maximum to minimum standardization. The formula is as follows:

(6) $$\begin{array}{c} x{}^{\prime }=\frac{x-\min A}{\max A-\min A}. \end{array}$$

The article "A BP Neural Network Algorithm for Multimedia Data Monitoring of Air Particulate Matter" was published in 2022. Journal: Comput Intell Neurosci.

## 4. Experimental Analysis

The neural network model construction, training, and testing of air particulate matter PM_2.5_ and PM_10_ are realized through the neural net package of *R* language. The original data of PM_2.5_ and PM_10_ and the four indexes of temperature and humidity collected by the light scattering sensor of the air detection equipment installed near the state control point of Yushan Park in Yuyao are used as the characteristic values [22], and the PM_2.5_ and PM_10_ indexes released by the state control point in Yuyao are used as the characteristic labels for model training. The real monitoring values of PM_2.5_ and PM_10_ are shown in Tables 1 and 2.

Furthermore, in order to objectively compare the prediction accuracy of the two models from the data, this study compares the prediction results of the two prediction models through four performance indexes: root mean square error (RMSE), average absolute error (MAE), average absolute error percentage (MAPE), and absolute error percentage (APE). The formulas of the four performance indexes are as follows:

(7) $$\begin{array}{c} \text{RMSE}=\sqrt{\frac{1}{n}\sum_{i=1}^{n}{\left|t_{i-}y_{i}\right|}^{2}},\\ \text{MAE}=\frac{1}{n}\left(\sum_{i=1}^{n}\left|t_{i}-y_{i}\right|\right),\\ \text{MAPE}=\frac{1}{n}\left(\sum_{i=1}^{n}\frac{t_{i}-y_{i}}{t_{i}}\right)100\%,\\ \text{APE}=\frac{\left|t_{i}-y_{i}\right|}{t_{i}}100\%, \end{array}$$

where *n* is the number of layers, *t*_*i*_ is the level of nodes, and *y*_*i*_ is the hourly average.

The trained neural network model is used to test the test data. From August 6, 2018, to August 12, 2018 (the data of the state control point of Yuyao Longshan park provided by Yuyao environmental protection bureau is used as a reference in this time period), the test comparison results of PM_10_ and PM_2.5_ with the state control point are shown in Figures 4 and 5, respectively [23, 24].

## 5. Conclusion

Due to the large difference in the value range of training data, the training time increases, resulting in inability to converge. In this experiment, the data are normalized by using BP neural network algorithm. After normalization, the training time is greatly shortened and convergence is achieved. It can be seen that normalization of data is particularly important for neural network. At the same time, the optimal neural network model is found by traversing the number of layers of hidden layer and the number of nodes of single layer. The trend and consistency of the two curves generated by the data calibrated by the model and the data of national control points are good, and the expected effect is achieved. Through experiments, it is verified that the air particulate matter calibration model based on the light scattering method and improved BP neural network algorithm has certain practicability and effectiveness. This air particulate matter monitoring method calibrated by software is a low-cost large-scale grid deployment to clarify the trend and diffusion law of air pollution, so as to determine the source of pollutants and reduce the scope of pollutants. It provides a feasible basis for full coverage, scientific analysis, and efficient management of hotspots in the regulatory area.

The article "A BP Neural Network Algorithm for Multimedia Data Monitoring of Air Particulate Matter" was published in 2022. Journal: Comput Intell Neurosci.

The prediction period studied in this paper is the next day. Because the time interval of all the data collected in this study is one day, the prediction can only be carried out for the city in one day. If the PM_2.5_ concentration can be predicted in a smaller time unit (such as hour), it will certainly be of better help to people's prevention work. With the enrichment and improvement of detailed data in the future, the amount of training data of neural network model will be doubled, which is bound to be conducive to the further training and prediction of the neural network model.

## Figures and Tables

**Figure 1:** The generation of PM_2.5_.

**Figure 2:** Physiological structure of neurons.

**Figure 3:** Activation function based on the basic structure of artificial neuron.

**Figure 4:** Comparison curve between PM_10_ model calibration value and national control points.

**Figure 5:** Comparison curve between PM_2.5_ model calibration value and national control points.

**Table 1:** Predicted and real monitored PM_2.5_ concentration values.

Serial number	Real monitoring value	Model predicted value
1	35	31.10972.526
2	62	57.84564512
3	50	54.23105623
4	45	40.89423561
5	33	43.56235871
…	…	
120	24	36.80122783
121	2.5	30.31336950
122	48	30.9870.3742
123	54	58.77795235
124	62	51.92018032

**Table 2:** Description of model construction.

Model input layer	4 nodes PM_2.5_PM_10_ humidity and temperature
Model hidden layer	The maximum number of layers is 2, and the maximum number of nodes in each layer is 10
Model output layer	1 node PM_2.5_
Model bias quantity	1
Model training data	The hourly average data of air monitoring equipment and state control points are randomly selected at a ratio of 0.9
Model test data	Hourly average data of air monitoring equipment and state control points with the remaining ratio of 0.1
Test evaluation function	According to the MSE evaluation standard of mean square error function, the optimal model of hidden layer is selected
Validation data	Hourly average data of air monitoring equipment and state control points

The article "A BP Neural Network Algorithm for Multimedia Data Monitoring of Air Particulate Matter" was published in 2022. Journal: Comput Intell Neurosci.

## Data Availability

The data used to support the findings of this study are available from the corresponding author upon request.
